# Surface Electromyography as a Method for Diagnosing Muscle Function in Patients with Congenital Maxillofacial Abnormalities

**DOI:** 10.1155/2020/8846920

**Published:** 2020-09-15

**Authors:** Liliana Szyszka-Sommerfeld, Mariusz Lipski, Krzysztof Woźniak

**Affiliations:** ^1^Department of Orthodontics, Pomeranian Medical University in Szczecin, Al. Powstańców Wlkp. 72, 70111 Szczecin, Poland; ^2^Department of Preclinical Conservative Dentistry and Preclinical Endodontics, Pomeranian Medical University in Szczecin, Al. Powstańców Wlkp. 72, 70111 Szczecin, Poland

## Abstract

Electromyography (EMG) is the most objective and reliable method available for imaging muscle function and efficiency, which is done by identifying their electrical potentials. In global surface electromyography (sEMG), surface electrodes are located on the surface of the skin, and it detects superimposed motor unit action potentials from many muscle fibers. sEMG is widely used in orthodontics and maxillofacial orthopaedics to diagnose and treat temporomandibular disorders (TMD) in patients, assess stomatognathic system dysfunctions in patients with malocclusions, and monitor orthodontic therapies. Information regarding muscle sEMG activity in subjects with congenital maxillofacial abnormalities is limited. For this reason, the aim of this review is to discuss the usefulness of surface electromyography as a method for diagnosing muscle function in patients with congenital malformations of the maxillofacial region. Original papers on this subject, published in English between 1995 until 2020, are located in the MEDLINE/PubMed database.

## 1. Introduction

Electromyography (EMG) is the most objective and reliable method available for imaging muscle function and efficiency, which is done by identifying their electrical potentials [1]. Electromyography takes two forms, i.e., intramuscular and global (surface electromyography, sEMG), depending on the way the electrodes are applied. In the case of intramuscular EMG, a needle and fine-wire electrodes are inserted into muscle tissue through the skin, whereas in global EMG surface electrodes are located on the surface of the skin. Moreover, another difference between these two approaches lies in the fact that intramuscular EMG detects single motor unit potential (motor unit action potential (MUAP)), while surface electromyography identifies superimposed MUAPs from many muscle fibers. As these signals include a weighted summation of the spatial and temporalis activity of many motor units, the analysis of sEMG recordings is limited to general muscle activity, cooperation between different muscles, and variability in their activity over time [1]. Another disadvantage of surface electromyography is its sensitivity to imbalances in impedance, and this may reduce the accuracy of EMG recordings and, as a consequence, result in low reproducibility. To ensure the reproducibility of this method, the interelectrode distance should be fixed, and a standard procedure for positioning the electrodes should be used to exclude variability in electrode placement [2–4]. The inconsistency in the impedance and reliability of sEMG could also be solved through normalization, which is the basic component of the data analysis. The normalization process is important for the preliminary processing of raw values to ensure further analysis. The standardized data provide information on the impact of occlusion on neuromuscular activity and ensure removal most of biological and technical noise, such as anatomical variations, skin, and electrode impedance. The process of normalizing the EMG results entails converting them into quotient indices. In this way, muscle electrical activity could be presented as a percentage of another high-reproducible activity of this muscle recorded under the same conditions, such as maximum voluntary contraction (MVC) (%MVC). The other possibility of quantitative analysis is to relate the electrical potentials of the muscles to the reference values obtained from the EMG measurements performed in the submaximal voluntary contraction (subMVC) [5, 6]. The undoubted advantage of global electromyography that compensates for the abovementioned limitations is its noninvasiveness [1]. Due to the simplicity of this method, its safeness, and availability, it has been used in studies on children [7–9].

The methodology of sEMG recordings, including electrode placement, EMG signal processing, and modelling, is based on the Surface Electromyography for Non-Invasive Assessment of Muscles (SENIAM) and The International Society of Electromyography and Kinesiology (ISEK) recommendations [1].

Masseter and anterior temporalis muscles are the muscles most frequently evaluated by sEMG. Masticatory muscle electrical activity can be assessed during static tests (rest, maximum, or sub-maximum voluntary clenching) or during active tests, such as opening or closing the mouth, protrusion, retrusion, lateral deviation of the mandible, chewing, swallowing, or speaking [1]. Rest activity is one of the most important static activities analysed. There is no isoelectric line observed in the sEMG recordings in this position determined by freeway space. However, some research has shown that the clinical rest position is an active muscle position because of the tone of the muscles involved in it [10]. Another important static test, which is frequently analysed, is maximum voluntary contraction (MVC). The EMG recordings during isometric contraction can be performed while clenching the teeth as hard as possible for 3 to 5 seconds, usually in an intercuspal position or during maximum clenching with a control substance, i.e., with cotton rolls placed on the mandibular second premolar and molars [11, 12]. EMG muscle potentials should also be evaluated in a fatigue test, which involves a continuous 10-second sub-maximum or maximum isometric muscle contraction. Median power frequency (MPF) and time-frequency distributions are the most objective and reliable EMG parameters for evaluating muscle resistance to fatigue [1]. In turn, the most frequent dynamic activity analysed by sEMG is mastication. It is usually expressed by such parameters as the duration of the masticatory act, the number of cycles, and its effectiveness depending on the forces generated and food consistency [13]. The use of electromyographic indices, such as the activity index (Ac), symmetry (percentage overlapping coefficient (POC), and torque coefficient (To, Tc)), makes it possible to assess the activity, coordination, and symmetry of the homologous, synergistic, and antagonistic muscles [1].

According to the literature, surface electromyography is widely used in orthodontics and maxillofacial orthopaedics to help diagnose and treat patients with temporomandibular disorders (TMD), as well as to assess stomatognathic system dysfunctions in patients with malocclusions or monitor orthodontic therapies [8, 14–22]. Information regarding muscle sEMG activity in subjects with congenital maxillofacial abnormalities is limited. For this reason, the aim of this review is to discuss the usefulness of surface electromyography as a method for diagnosing muscle function in patients with congenital malformations of the maxillofacial area. Patients with these abnormalities often suffer from aesthetic, morphological, and functional problems in the dentofacial region. Congenital maxillofacial defects have significant psychological and socioeconomic effects on a patient's quality of life and require a multidisciplinary team approach if it is to be managed properly. Clefts of the lip, alveolus, and/or palate are the most frequent head and neck congenital deformities that significantly affect the functions of the stomatognathic system and disrupt normal facial structure [7, 9].

## 2. Material and Methods

Original peer-reviewed papers on this subject, published in English between 1995 until 2020, are located in the MEDLINE/PubMed database. The literature search strategy was conducted as follows: keyword “surface electromyography” was combined with each of “congenital maxillofacial abnormalities,” “cleft lip and palate,” “Down syndrome,” “hemifacial microsomia,” “craniosynostosis.”

### 2.1. Imaging of Muscle Function in Cleft Lip and Palate (CLP) Patients by means of sEMG

Clefts of the lip, alveolus, and/or palate are the most frequent congenital facial malformations that significantly affect the functions of the stomatognathic system and disrupt dentofacial aesthetics [23, 24]. Besides dysfunctional facial expressions, patients with cleft lip and palate may have serious functional problems with sucking, swallowing, breathing, chewing, speaking, hearing, and social integration [25, 26]. Abnormal jaw growth in CLP patients can result in severe malocclusion, which in turn may affect the functioning of the maxillofacial muscles [7]. Successful treatment of a cleft patient involves multidisciplinary surgical and nonsurgical care performed from birth through to adulthood [27]. In a few published studies, surface electromyography was used to detect the electrical potentials of the superior orbicularis oris muscle and masticatory muscles in cleft lip and palate patients [7, 9, 28–33].

In a study by Szyszka-Sommerfeld et al. [9], the authors analysed the electrical activity of the superior orbicularis oris muscle by means of sEMG in patients ranging in age from 6 to 13 years. Their study cohort comprised 45 children operated on for unilateral complete cleft lips and palates (UCCLP). They were compared with 40 control subjects with no cleft lip and palate. Electromyographical recordings were taken in the rest position and during saliva swallowing, lip protrusion, and reciprocal compression of the lips, as well as while producing the bilabial phonemes /p/, /b/, and /m/ associated with the vowel /a/. The authors observed that patients with unilateral repaired complete cleft lip and palate have abnormal upper lip function characterized by higher EMG activity of the superior orbicularis oris muscle during saliva swallowing and reciprocal compression of the lips in the cleft group. Thus, they suggested that the excessive force applied by a repaired cleft lip to underlying structures during saliva swallowing and lip compression may affect facial morphology. Furthermore, the authors observed that EMG values at rest and when producing the bilabial phonemes /p/, /b/, and /m/ combined with the vowel /a/ were comparable in both groups.

Ravera et al. [28] assessed superior orbicularis oris muscle function at rest, during saliva swallowing, speaking, chewing, and apple swallowing in 14 children operated on for unilateral CLP and ranging in age from 6 to 12 years. All cleft patients had clinically short upper lips, abnormal lip seal, and inhibited sagittal development of the midface. The control group included 14 noncleft children aged between 8 and 11 years. The authors noted significantly higher results for the electrical potentials of the superior orbicularis oris muscle at rest and during saliva swallowing in the cleft group, while EMG activity levels during speech were similar in both cleft and noncleft subjects. They stated that the higher electrical activity of the upper lip at rest and during swallowing of saliva in children with CLP suggests that upon higher functional demands their activity increases less than that in noncleft children. They also suggested that greater electrical potentials of the superior orbicularis oris muscle reflects increased force on the maxilla and as a consequence, the surgical treatment of cleft lip has an iatrogenic effect on facial growth.

Szyszka-Sommerfeld et al. [7] analysed masticatory muscle activity by means of sEMG in children surgically treated for unilateral complete cleft lip and palate. The authors also assessed the possible factors associated with such EMG activity. The study population included 82 children with mixed dentition and Class I occlusions. The cleft group consisted of 25 children aged between 6 and 13 years. They were compared with 57 control subjects aged between 6 and 12 years with no cleft lip and palate. The EMG recordings of the temporalis and masseter muscles were performed at rest and during maximum voluntary contraction (MVC). Their results showed that children with UCCLP had altered temporalis muscle function at rest compared with noncleft subjects. They also found that the presence of malocclusion, such as posterior crossbite, affects the temporalis muscle activity in cleft patients. The authors declared that early diagnosis and orthodontic treatment of malocclusions are necessary to achieve the correct occlusion and improvement in muscle function in these patients.

da Costa et al. [29] used sEMG to analyse masticatory muscle function at rest and during isometry and mastication in 33 children with complete cleft lip and palate as well as in 33 noncleft patients aged between 6 and 12 years. They found much higher EMG potentials of the temporalis and masseter muscles in cleft subjects at rest and during inactive period of mastication, whereas electrical activity in the left masseter muscle and temporalis muscles during active period of mastication and in every muscle during isometry was significantly lower. The authors also observed that the muscles of cleft children remained active for longer than in patients with no cleft. da Costa et al. suggested that the higher length of the chewing cycle in the cleft group might be a consequence of malocclusion and might result in functional inefficiency, making mastication more difficult.

Li et al. [30] evaluated masticatory muscle function in 29 patients aged from 11 and 21 years with unilateral cleft lip and palate (UCLP) and anterior crossbite. The control group consisted of 28 noncleft subjects with normal occlusion. They observed that the temporalis muscle EMG potentials at rest were significantly higher in UCLP patients compared to the controls. The results of their study also showed altered masseter muscle function at rest and significantly lower masseter muscle electrical activity during maximum clenching in the intercuspid position in the cleft group.

Surface electromyography was also used to image masticatory muscle function in cleft lip and palate subjects with pain-related temporomandibular disorders (TMDs) [31, 32]. TMDs are a collective term associated with a number of clinical conditions that affect the masticatory muscles, the temporomandibular joint (TMJ), and associated structures. The main signs and symptoms of TMDs are muscle and joint sensitivity or pain, joint noises, and derangements in the movements of the mandible [34–36]. Patients with clefts are potentially at risk of developing TMD, due to psychosocial burdens and malocclusions predisposing them to this disorder [37].

Szyszka-Sommerfeld et al. [31] evaluated temporalis and masseter EMG activity in 31 CLP patients with pain-related TMD and 32 CLP subjects with no TMD aged between 6 and 14 years. They observed that masticatory muscle activity at rest in pain-related TMD cleft subjects was significantly higher and masticatory muscle EMG potentials during maximum voluntary clenching were markedly lower than those in cleft children with no TMD diagnosis. Moreover, they found a significant increase in the Asymmetry Index for temporalis and masseter muscle rest activity in pain-related TMD patients. The authors concluded that cleft children diagnosed with pain-related TMD have altered masticatory muscle activity, and this can affect their muscle function.

In another study by Szyszka-Sommerfeld et al. [32], the authors analysed the diagnostic efficiency of sEMG in identifying CLP subjects with temporomandibular disorders. Their sample comprised 88 patients with cleft lip and palate and mixed dentition. The study population was subdivided into three groups: a pain-free TMD group, a TMD-pain group, and a non-TMD group. The electrical activity of the temporalis and masseter muscles was assessed in the rest position and during maximum voluntary contraction. The results of the study revealed that surface electromyography is diagnostically useful in recognition of CLP patients with pain-related TMD and it could be used as an adjunctive tool in the identification of this disorder. They found that the highest diagnostic efficiency of sEMG in terms of identifying subjects with TMD and pain-related TMD was observed for the mean values of temporalis and masseter muscle activity as well as the Asymmetry Index of the masseter muscles in a rest position.

sEMG was also used to detect muscle electrical potentials while monitoring orthodontic or surgical therapies in cleft lip and palate patients. Sabbag et al. [33] assessed the EMG activity of the masseter and temporalis muscles in 32 nonsyndromic complete unilateral CLP patients surgically treated with 2 different palate repair protocols (one-stage vs. two-stage). The EMG potentials of the masticatory muscles were recorded at rest and during chewing. The authors observed similar masseter and temporalis EMG activity while mastication and at rest after one- and two-stage palate closure.

### 2.2. Assessment of Muscle Function in Patients with Down Syndrome (DS) by means of sEMG

Down syndrome is a chromosomal alteration caused by trisomy 21. Many comorbidities are associated with DS, including obstructive sleep apnea and masticatory muscle alteration. One of the characteristics most commonly found in patients with Down syndrome is the presence of generalized muscular hypotonia, particularly of the masticatory and oropharyngeal muscles, which directly affect the stomatognathic system, resulting in speech, swallowing, and mastication impairments in these individuals [38, 39]. Few studies have assessed muscle activity in DS patients by means of sEMG. In a published paper, sEMG was used to evaluate masticatory muscle function while monitoring orthodontic therapy in subjects with Down syndrome [39, 40].

Giannasi et al. [39] assessed the therapeutic effects of surface neuromuscular electrical stimulation, mastication apparatus, and a mandibular advancement device with an embedded thermosensitive microchip on masticatory muscle function, physiological sleep variables, and salivary parameters in patients with Down syndrome aged between 18 and 40 years. sEMG was used to detect temporalis and masseter muscle electrical potentials. Following an analysis of the study results, the authors stated that the primary outcomes would be an improvement and/or reestablishment of masticatory muscle function and physiological sleep variables in these target subjects since patients with DS commonly exhibit generalized muscular hypotonia and dysfunction of the oropharyngeal musculature.

Mazille et al. [40] used video and sEMG recordings to investigate the therapeutic impact of wearing an orthetic intra-oral appliance on chewing variables in 8 Down syndrome subjects with a mean age 27 ± 6 years. The simultaneous use of EMG and video recordings revealed the presence of lower jaw movements not corresponding to EMG activities in the masticatory muscles. The authors observed that, compared to the pretreatment state, wearing an occlusal appliance lowered chewing frequency and increased masticatory time.

### 2.3. sEMG Recordings of Patients with Other Congenital Maxillofacial Abnormalities

Surface electromyography also provided the basis for assessing masticatory muscle activity in patients with other congenital maxillofacial anomalies, such as hemifacial microsomia or craniosynostosis [41–43]. Hemifacial microsomia is the second most common congenital anomaly of the craniofacial region behind cleft lip and palate. This malformation is characterized by asymmetric facial growth with mandibular and muscle involvement. It primarily affects the ear, mouth, and jaw areas, though it may also involve the eye, cheek, neck, and other parts of the skull, as well as nerves and soft tissue [44]. Craniosynostosis is a developmental craniofacial malformation, resulting in impairment of brain development and abnormally shaped skull. The main cause of craniosynostosis is premature closure of one or more cranial sutures. When left untreated, craniosynostosis can cause serious complications, such as impairment of mental development, facial abnormality, sensory, respiratory and neurological dysfunction, anomalies affecting the eye, psychological disturbances, sleeping impairment, and eating difficulties [45].

Telich-Tarriba et al. [41] used sEMG to assess masticatory muscle function in patients with hemifacial microsomia (HFM). They compared the bite force and electrical activity of masseter muscle in 20 children with hemifacial microsomia and 10 healthy controls with a mean age of 7.2 years. EMG recordings were performed in maximum intercuspation and at rest from both sides of the face. The authors found that masseter muscle EMG potentials in maximum intercuspation were significantly lower in HFM patients compared with both the healthy side and the control group. Moreover, they observed significant differences in the masseter muscle EMG activity of affected and nonaffected sides at rest in children with hemifacial microsomia.

Suzuki et al. [42] investigated the relationship between mandibular ramus height and masticatory muscle function in 29 patients with hemifacial microsomia. They observed that decreased mandibular ramus height was significantly correlated with both reduced masseter muscle EMG potentials and the amount of mandibular lateral deviation at the time of maximum opening on the affected side. The authors suggested that decreased mandibular ramus height may cause dysfunction of the masseter muscles but not the temporalis muscle on the affected side in patients with hemifacial microsomia.

Martini et al. [43] analysed masticatory muscle function in 15 patients with craniosynostosis after cranioplasty, as well as in 25 7-year old nonoperative healthy controls. The maximum bite force and EMG activity of the temporalis and masseter muscles were assessed. The results of the study revealed that the EMG potentials of the temporalis muscle correlated positively with the bite force and showed a slightly lower resting activity in the control group, whereas muscle fatigue occurred slightly faster in both muscles of children who had been operated on, but no statistically significant differences between the two groups were observed.

## 3. Conclusions

This literature review of studies involving surface electromyography demonstrated its usefulness as a method of muscle function imaging in patients with congenital abnormalities of the maxillofacial region. sEMG could be used as an additional tool in the diagnosis or monitoring orthodontic therapies in these patients, thereby expanding our knowledge about the anatomy, physiology, and pathology of their stomatognathic system.

In the years 1995–2020, only a few papers were published that examined the possibilities of using surface electromyography in diagnosing muscle function in subjects with developmental maxillofacial anomalies. This is probably mainly due to the difficulties involved in selecting the study population. Moreover, among the presented papers, only some studies included sufficiently large study groups as well as sEMG signal normalization. For these reasons, further expanded investigations on the subject would be needed.
